The article "Network Anomaly Traffic Detection Algorithm Based on RIC-SC-DeCN" was published in 2022. Journal: Comput Intell Neurosci.

# Network Anomaly Traffic Detection Algorithm Based on RIC-SC-DeCN

**DOI:** 10.1155/2022/8315442

**Published:** 2022-05-24

**Authors:** Xingyu Gong, Ke Cao, Na Li, Pengtao Jia

**Affiliations:** College of Computer Science and Technology, Xi'an University of Science and Technology, Xi'an 710054, China

## Abstract

In the research of network abnormal traffic detection, in view of the characteristics of high dimensionality and redundancy in traffic data and the loss of original information caused by the pooling operation in the convolutional neural network, which leads to the problem of unsatisfactory detection effect, this paper proposes a network abnormal traffic detection algorithm based on RIC-SC-DeCN to improve the above problems. Firstly, a recursive information correlation (RIC) feature selection mechanism is proposed, which reduces data redundancy through the maximum information correlation feature selection algorithm and recursive feature elimination method. Secondly, a skip-connected deconvolutional neural network model (SC-DeCN) is proposed to reduce the information loss by reconstructing the input signal. Finally, the RIC mechanism and the SC-DeCN model are merged to form a network abnormal traffic detection algorithm based on RIC-SC-DeCN. The experimental results on the CIC-IDS-2017 dataset show that the RIC feature selection mechanism proposed in this paper has the highest accuracy when using MSCNN as the detection model compared to the other three, which can reach 96.22%. Compared with the other five models, the SC-DeCN model has the highest detection accuracy, while the model training time is moderate and can reach 96.55%. Compared with the SC-DeCN model, the RIC-SC-DeCN model reduces the overall training time by 45.50%, while the accuracy rate is increased to 97.68%. It shows that the algorithm proposed in this paper has a good detection effect in the detection of network abnormal traffic.

## 1. Introduction

With the increasing development of computer networks, the Internet has been integrated into all aspects of people's lives. Shopping, medical [1], communication [2], and other aspects of data are also transmitted and interacted through the network. At the same time, network security incidents occur frequently, and various network attacks often cause abnormal changes in network traffic. The network abnormal traffic detection technology proposed to solve the above network security problems is one of the important means to ensure network security.

In the detection of network abnormal traffic, the network traffic data attack forms are diverse and have the problem of noise feature. Therefore, reasonable feature selection for data can not only reduce the resource consumption of processing, storing, and transmitting data but also improve the accuracy of anomaly detection [3, 4]. In recent years, many scholars have conducted in-depth research on the feature selection of network traffic data. The study in [5] uses the chi-square test for feature selection, which can effectively handle high-dimensional data of network traffic. The work in [6] proposes an adaptive binning feature selection algorithm based on information gain for the problem of long training and detection time for anomaly detection systems based on deep learning. The research in [7] proposes a random forest algorithm based on recursive feature elimination (RFE-RF) to address the low accuracy of high-dimensional data in classification tasks.

In addition, in the detection of network abnormal traffic, the pooling operation in the convolutional neural network used can easily lead to the loss of original feature information [8, 9]. In response to this problem, [10] proposes a deep convolutional neural network model based on deconvolution feature extraction, which can automatically extract rich implicit features from bottom-level boundaries to high-level objects. The work in [11] proposes an improved one-dimensional convolutional neural network, which removes the pooling operation in the convolutional neural network and preserves the complete traffic information as much as possible. However, this will slow down the feature extraction and the network. The training time of the model also becomes longer.

For the feature selection problem mentioned above, the research in [5, 6] excessively removes redundant information and reduces the detection accuracy, and the work in [7] has a high computational cost for feature selection. In addition, for the information loss problem, the network anomaly detection algorithm proposed in [10, 11] improves the information loss problem, but the disadvantage is that the training time of the model becomes longer. In view of the above-mentioned problems of unsatisfactory feature selection and information loss, this paper proposes a network abnormal traffic detection algorithm based on RIC-SC-DeCN. Firstly, for the problem of data redundancy and high dimensionality, a RIC feature selection mechanism is proposed, which reduces data redundancy through the maximum information correlation feature selection algorithm and recursive feature elimination method. Secondly, aiming at the problem of information loss of network traffic data, a SC-DeCN model is proposed, which combines the deconvolutional neural network to reconstruct the input signal to reduce the information loss. Finally, the RIC mechanism and the SC-DeCN model are merged to form a network abnormal traffic detection algorithm based on RIC-SC-DeCN. Our contributions are as follows:

1. A RIC feature selection mechanism is proposed. Through the maximum information correlation feature selection algorithm and recursive feature elimination method to reduce data redundancy, network traffic features can be extracted more efficiently.
2. A SC-DeCN model is proposed. The combination of shallow convolutional neural network information and deep deconvolutional neural network information makes feature extraction more accurate, thereby reducing information loss.
3. Combine the proposed RIC feature selection mechanism with the SC-DeCN model to form a network abnormal traffic detection algorithm based on RIC-SC-DeCN. Compared with other classification algorithms, the method proposed in this paper can greatly reduce the training time of the model and improve the accuracy of anomaly detection.

The remainder of this paper is organized as follows.  Section 2 introduces the work related to network abnormal traffic detection; Section 3 mainly describes the RIC-SC-DeCN algorithm; Section 4 introduces the experimental dataset, and describes the experimental results and analysis in detail; the conclusion and future work part are in Section 5.

## 2. Related Work

Feature selection techniques have been widely used in many fields. Among them, in the detection of network abnormal traffic, many scholars use feature selection methods to reduce high-dimensional to low-dimensional data, thereby reducing the time for model training and detection. Aiming at the multiobjective feature selection problem in intrusion detection systems, Zhu et al. [12] proposed a population evolution strategy based on a special control method and predefined multiobjective search, which can distinguish anomaly types. Zhao et al. [13] considered the redundancy between features and the influence between features and classes and proposed a new Redundancy Penalized Feature Mutual Information Algorithm (RPFMI). Sumaiya Thaseen et al. [14] utilized chi-square feature selection and an ensemble of Support Vector Machines (SVM), Modified Naive Bayes (MNB), and LP Boost classifiers to build an intrusion detection model. Ran [15] proposed an MRMR-based network traffic feature selection method, which reduced the dimension of network traffic data. However, none of the methods proposed above make a reasonable feature selection for network traffic datasets. Redundant features will be removed excessively, resulting in the loss of important information.

Deep learning models have powerful feature extraction capabilities and do not require expensive manual feature engineering, so they are widely used in network abnormal traffic detection tasks. Aceto et al. [16] designed a traffic classifier based on automatically extracted features, using deep learning as a feasible strategy for network abnormal traffic detection. Erxue [17] utilizes word embeddings and text convolutional neural networks to extract effective information from the payload, synthesizes statistical features and payload features, and proposes a new TR-IDS intrusion detection system.

Due to the powerful feature capturing capabilities of convolutional neural networks, many scholars have conducted in-depth research and proposed various variants [18–21]. Basumallik et al. [18] improved a convolutional neural network to identify vulnerable points in PMU networks. Zhang et al. [19] proposed a fraud detection model based on convolutional neural networks, which constructed an input feature ranking layer to reorganize the original transaction features to form different convolutional patterns. Gu et al. [20] proposed an improved bidirectional linear convolutional neural network model. In order to improve the performance of network intrusion detection, Tian et al. [21] adopted the method of Faster Regional Convolutional Neural Network (Faster R-CNN) to complete network anomaly detection.

In addition, there are many research works that integrate different types of neural networks to improve the accuracy of network abnormal traffic detection [22, 23]. Kim and Cho [22] proposed a network abnormal traffic detection method based on a hybrid algorithm of convolutional neural network and long-short-term memory network, using a combination of CNN and LSTM to learn and classify traffic packets in time and space, preserving the order of feature sequences characteristics to more accurately identify network traffic with hierarchical spatiotemporal characteristics. Ding and Peng [23] proposed a multilayer network structure CNN algorithm to convert the network traffic data in KDD99 into data that can be input by a convolutional neural network. Convolution kernels of different scales are used to extract different levels of features from a large number of high-dimensional unlabeled raw data, which greatly improves the classification performance. Javed et al. [24] proposed a convolutional neural network with a multistage attention mechanism that converts data traffic into vectors for anomaly detection. Experimental results show that the proposed method achieves good performance on both single-source and mixed multisource anomaly types. Khan et al. [25] proposed a new deep learning model (TSDL) that introduced a low-cost DSAE method that is able to learn useful feature representations from large amounts of unlabeled data and automatically and efficiently sort.

## 3. Network Anomaly Traffic Detection Algorithm

This section provides an overview of our proposed feature selection mechanism and neural network model, which is the main part of this paper.

### 3.1. The Overall Framework of Network Anomaly Traffic Detection Algorithm

The overall framework of the RIC-SC-DeCN network abnormal traffic detection algorithm proposed in this paper is shown in Figure 1. The algorithm includes three modules: data preprocessing, feature selection, and abnormal detection. The main task of the data preprocessing module is to standardize the features and one-hot encoding the labels and input the processed data to the feature selection module. In the feature selection module, the RIC feature selection mechanism is adopted. Firstly, remove features with zero variance; Second, use the feature selection with maximum information correlation and select some features with the best phenotype according to the correlation between the feature and the phenotype. Finally, the optimal feature subset is selected by recursive feature elimination method, and the feature subset is input to the anomaly detection module. The anomaly detection module inputs the optimal feature subset into the convolutional neural network to automatically learn the traffic features and then deconvolutes the deep information of the convolutional, through fusing the shallow information in the convolutional neural network with the deep information in the deconvolutional neural network, the SC-DeCN model is constructed, and the network abnormal traffic is detected by this model.

## 4. RIC Feature Selection Mechanism

For the problem that most network traffic data is high-dimensional and accompanied by noise, this paper proposes a feature selection mechanism of Recursive Information Correlated (RIC), which extracts key features from the original network traffic data and reduces the impact of noise features on network abnormal traffic detection. The RIC feature selection mechanism includes three steps: first, removing irrelevant features; second, performing feature selection with maximum information correlation; finally, using recursive feature elimination to select features.

### 4.1. Remove Irrelevant Features

The network traffic dataset contains features with a variance of 0, and these features have no effect on judging whether the network traffic is abnormal. Therefore, these irrelevant features should be removed. Given a network traffic data *x*, the network traffic feature is used to *f* represent, and the network traffic feature set is used to *S* represent, then the expressions of features sets *S* and feature *f* are shown in the following:

(1) $$\begin{array}{c} S=\left\{f_{1},f_{2},f_{3},\cdots ,f_{b}\right\}, \end{array}$$

(2) $$\begin{array}{c} f=\left\{x_{1},x_{2},x_{3},\cdots ,x_{m}\right\}. \end{array}$$

Here, *f*_*b*_ represents the *b* dimension feature in the network traffic dataset, *x*_*m*_ represents *m* pieces of network traffic data, and the feature set after removing irrelevant features is *S*1={*f*_1_, *f*_2_, *f*_3_, ⋯, *f*_*d*_, *d* < =*b*}.

### 4.2. Feature Selection of Maximum Information Correlation

According to the correlation between the feature and the label, select the *t* features that are most related to the label and delete the features that are not related to the label. Use the idea of an F-test to select the *t* features with the most correlated features and labels. The method is to calculate the *F* value of each feature, query the *F* distribution table, and select the *t* features that are most relevant to the type of network traffic attack.

There are *k* kinds of attacks on the network traffic data, the network data of the *j* attack type is *n*_*j*_, and the expression of the average value $\bar{x}$ of the network traffic data is as follows:

(3) $$\begin{array}{c} \bar{x}=\frac{\sum_{j=1}^{k}\sum_{i=1}^{n_{j}}x_{ij}}{n}. \end{array}$$

Here *x*_*ij*_ represents the *i* network traffic data of the *j* label type and *n* is the total number of network traffic data. The sum of the squares of the overall differences of all attack types of network traffic data *SST* is expressed as follows:

(4) $$\begin{array}{c} SST=\sum_{j=1}^{k}\sum_{i=1}^{n_{j}}{\left(x_{ij}-\bar{x}\right)}^{2}. \end{array}$$

The sum of squares of differences within each attack type of network traffic data *SSE* is expressed as follows:

(5) $$\begin{array}{c} SSE=\sum_{j=1}^{k}\sum_{i=1}^{n_{j}}{\left(x_{ij}-\bar{x_{j}}\right)}^{2}. \end{array}$$

Here, $\bar{x_{j}}$ represents the mean value of the *j* class label, as follows:

(6) $$\begin{array}{c} \bar{x_{j}}=\frac{\sum_{i=1}^{n_{j}}x_{ij}}{n_{j}}. \end{array}$$

The sum of squares of differences between attack types of network traffic data *SSB* is expressed as follows:

(7) $$\begin{array}{c} SSB=SST-SSE\\ =\sum_{j=1}^{k}n_{j}{\left(\bar{x_{j}}-\bar{x}\right)}^{2}. \end{array}$$

The expression of the correlation function *F*(*t*) between the feature of the network traffic data and the attack type is the ratio of the intraclass difference *MSB* and the interclass difference *MSE*, and *F*(*t*) is expressed as follows:

(8) $$\begin{array}{c} F\left(t\right)=\frac{MSB}{MSE}. \end{array}$$

The intraclass difference *MSB* is expressed as in (9), and the interclass difference *MSE* is expressed as in (10).

(9) $$\begin{array}{c} MSB=\frac{SSB}{k-1}, \end{array}$$

(10) $$\begin{array}{c} MSE=\frac{SSE}{n-k}. \end{array}$$

For a feature set *S*_1_ of network traffic, calculate the F-value of each feature and attack type. Select the *t* features most relevant to the attack type according to the F-test distribution table. After feature selection with maximum information correlation, the selected feature subset is *S*_2_={*f*_1_, *f*_2_, *f*_3_, ⋯, *f*_*t*_, *t*〈*d*}.

### 4.3. Recursive Feature Elimination

Recursive feature elimination is used to select the optimal feature subset, random forest (RF) is used as the classifier, each feature *X* and phenotype *Y* are trained, and the classifier is used to evaluate the influence of feature *X* on phenotype *Y*. Find the optimal dataset after multiple cross-validations. The optimal subset of features finally selected is *S*_3_={*f*_1_, *f*_2_, *f*_3_ … *f*_*h*_, *h*〈*t*}.

The RIC feature selection mechanism proposed in the paper includes three steps: Step 1, remove irrelevant features, remove those features whose feature columns are all zero or zero variance, and obtain feature subset *S*_1_; Step 2, carry out maximum information correlation feature selection, according to the correlation between features and phenotype, select the *t* features with the best phenotype, and obtain the feature subset *S*_2_; Step 3, use the recursive feature elimination method to select the optimal feature subset *S*_3_.

### 4.4. SC-DeCN Network Anomaly Traffic Detection Model

The convolutional neural network feature extraction process focuses on the distribution of data information, which can effectively distinguish normal and abnormal data distribution and is widely used in network abnormal traffic detection. However, in the process of pooling, it will cause a loss of original information. In order to solve this problem, the paper proposes a SC-DeCN model for network abnormal traffic detection. The model mainly consists of three parts: (1) A CNN module is designed, which mainly includes convolutional layers and pooling layers, and the main task is to automatically extract network traffic features from the optimal feature subset after feature selection. (2) A DeCN module is designed to deconvolute the deep information of the CNN module to extract richer feature information. (3) Combined with the shallow information of the CNN module and the deep information of the DeCN module, the SC-DeCN model is constructed to detect network abnormal traffic and determine which kind of attack the network abnormal traffic belongs to. The model diagram is shown in Figure 2.

(1) The 1st layer is the input layer, the input is network traffic data, and the input of the model is the 20-dimensional network traffic feature after feature selection.
(2) The 2nd and 3rd layers are convolutional layers. In traditional neural networks, different neurons between the two layers connect with each other, resulting in a large number of parameters to learn and bringing some difficulty in training. The convolutional layer has a local connection and weight sharing, which greatly reduces the number of parameters. The expression of convolution layer *a*_*i*_ is shown in the following equation:
  (11) $$\begin{array}{c} a_{i}=g\left(a_{i-1}*w_{i}+b_{i}\right). \end{array}$$
Among them, *w*_*i*_ is the weight of the convolution kernel of the *i* layer, *a*_*i*−1_ is the output of the convolution layer of the *i* − 1 layer, *b*_*i*_ is the bias vector of the *i* layer, *∗* is the convolution operation, and *g* is the activation function. Each layer in the convolution is top-down, and the expression of the shape feature *o* of the feature map is shown in the following:
  (12) $$\begin{array}{c} o=\left[\frac{c-e+2p}{s}\right]+1. \end{array}$$
The input feature map of the previous layer is *c*, the size of the convolution kernel is *e*, the stride is *s*, and the number of rows and columns filled with 0 in the feature shape is *p*.
(3) The 4th layer is the pooling layer, and the pooling window of the pooling layer is 2. The pooling layer is equivalent to further sampling the features and also reduces the dimension of the features. The expression of the pooling layer *h*_*j*_ is shown in the following equation:
  (13) $$\begin{array}{c} h_{j}=\beta_{j}\text{down}\left(h_{j-1}\right)+b_{j}. \end{array}$$
Here, *β*_*j*_ represents the activation value, “*do*  *wn*” represents downsampling, *h*_*j*−1_ is the output of the *j* − 1 layer of the pooling layer, and *b*_*j*_ represents the output of the *j* layer.
(4) The 5th, 6th, and 7th layers are deeper convolutional and pooling layers.
(5) Layers 8, 9, and 10 are deconvolution layers. Unlike the convolutional layer, its network signals are down-top and automatically use the deconvolution network to extract image high-level features, which can generally reflect the essence of the sample more than the original dataset. The expression of the shape feature *o*_2_ of the feature map in the deconvolution network is shown in the following equation:
  (14) $$\begin{array}{c} o_{2}=\left[\frac{c_{2}+2p_{2}-e_{2}-\left(e_{2}-1\right)*\left(l-1\right)}{s_{2}}\right]+1. \end{array}$$
The feature shape of the input feature map of the previous layer is *c*_2_, the size of the convolution kernel is *e*_2_, the step size is *s*_2_, *l* − 1 is the number of spaces inserted, and the number of rows and columns filled with 0 in the feature shape for *p*.
(6) The 11th layer combines the information of layer 4 and layer 10 as the input of layer 12 (Flatten layer). Combine the shallow features of convolutional neural networks with the deep features of deconvolutional neural networks.
(7) Layers 13 and 14 are fully connected layers with softmax layers, and the expression is shown in the following equation:
  (15) $$\begin{array}{c} y=\text{softmax}\left(w*o3+b\right). \end{array}$$

Among them, softmax represents the activation function, *w* represents the weight of the fully connected layer, *o*_3_ represents the feature map after connection through the skip level, *b* represents the bias of the fully connected layer, and the softmax layer classifies the network traffic data to determine whether the network traffic data belongs to what kind of attack.

Finally, the RIC feature selection mechanism in Section 3 and the SC-DeCN model in this section are combined to form the RIC-SC-DeCN network abnormal traffic detection algorithm in this paper.

## 5. Experimental Simulation Results and Analysis

The experimental operating system environment is Windows10, the computer hardware cup is i5-11260H, 16 GB memory, and it is programmed in Python 3.7 software environment.

### 5.1. Introduction and Analysis of Dataset

The CIC-IDS-2017 dataset is proposed by the Communications Security Establishment (CSE) & the Canadian Institute for Cybersecurity (CIC), covering all 11 necessary criteria for common security network events. The dataset contains normal traffic and 14 common attacks, and each record has 78 features. Because CIC-IDS-2017 does not divide the training set and test set, 80% and 20% are used to divide it into a training set and test set in this experiment. In addition, this ratio has been used by many researchers recently.

### 5.2. Data Preprocessing

The data set CIC-IDS-2017 contains a large number of outliers and missing values, which will cause the data model to lose a lot of useful information and make the rules contained in the model more difficult to grasp. Therefore, these data need to be processed before analysis and modeling.

(1) First, the outliers and missing values in the network traffic dataset are processed. Due to a large amount of data in the network traffic data set, the method adopted in this paper is to directly delete the data rows with null values and outliers.
(2) Converts the text type in each connection in the raw data to numeric form.
(3) Data standardization, the paper adopts the minimum and maximum normalization processing, which is a linear change of the original data, and maps the value to the [0, 1] interval. The conversion formula is in the following equation:
  (16) $$\begin{array}{c} x*=\frac{x-\text{min}}{\text{max}-\text{min}}, \end{array}$$
where max is the maximum value of the sample data, min is the minimum value of the sample data, and max − min is the extremely poor.
(4) One-hot encoding is performed on the label, because label data is an attack type of network traffic, which is a discrete type, does not have seriality, and cannot directly compare the size. Using one-hot encoding can better represent the relationship between labels.

### 5.3. Model Parameter Settings

After many experiments to adjust the parameters, this experiment selects the following hyperparameters for model training:

1. *Batch.* If the value of the batch is too small, the fast calculation will not be possible. On the contrary, the weights cannot be updated well, and the experimental results show that a batch of 256 works best.
2. *Epoch.* If the epoch is set too large, the network training will overfit, resulting in lower test accuracy. The experimental results show that an epoch of 4 has the best effect.
3. *Dropout.* In this experiment, the dropout is 0.5. The experiment effect is the best.

### 5.4. Evaluation Indicators

This experiment uses AR (Accuracy Rate), RR (Recall Rate), FAR (False Alarm Rate), F1-Score, and Time as indicators for performance evaluation. AR is used to evaluate the overall performance of the system, RR represents the ratio of anomaly examples detected by network anomaly traffic detection models, FAR is the ratio of misclassification, and F1-Score is a comprehensive indicator of precision and recall.

## 6. Experimental Results and Analysis

### 6.1. RIC Feature Selection Mechanism Experiment

In order to verify the effectiveness of the RIC feature selection mechanism proposed in this paper, the MSCNN model is used as the basic classification model, and the MIR mechanism, the RFE mechanism, the CHI mechanism, and the RIC mechanism proposed in this paper are used to select the features in the CIC-IDS-2017 dataset.

From Table 1, it can be concluded that the feature subsets selected by the four feature selection mechanisms are different. In the experiments in this section, the four feature subsets in Table 1 are used as input, and the MSCNN model is used for anomaly detection. The AR, RR, and F-Score of the above four feature selection mechanisms are shown in Figure 3, and the FAR is shown in Figure 4.

As can be seen from Figure 3, the feature subset selected by the RIC mechanism has the best performance in AR, RR, and F-Score on the MSCNN model compared to the MIR mechanism, the RFE mechanism, and the CHI mechanism. As can be seen from Figure 4, the FAR of the RIC mechanism on the CIC-IDS-2017 dataset is only 3.89%, which is 0.5% lower than that of the RFE mechanism, with the lowest FAR in the comparative experiment. The specific experimental data are shown in Table 2. In this table, select-time represents the time required for feature selection, Model-time represents the time required for model training, and Total-time represents the time required for feature selection and model training.

As can be seen from Table 2, compared with the MIR mechanism, the RIC mechanism improves AR, RR, and F-Score by 3.10%, 3.02%, and 3.11%, and the detection time increase is 49.71%. The RIC mechanism improves the AR, RR, and F-Score by 0.65%, 0.5%, and 0.61% compared with the RFE mechanism and shortens the time by 70.38%. The RIC mechanism improved AR, RR, and F-Score by 2.09%, 1.98%, and 2.09% compared with the CHI mechanism. The detection time increased by 46.93%.

Both the MIR mechanism and the CHI mechanism belong to the filtering feature selection method. The advantage of this method is that the computational cost of feature selection is short, and the time complexity is *T*(*n*)=*n*. The RFE mechanism should use the performance of the classifier as the evaluation criterion of the feature subset and traverse all possible combination feature subsets to select the optimal feature subset. The time complexity is *T*(*n*)=*n*^2^, and the computational cost of feature selection is relatively large, not suitable for large data samples. The time complexity of the RIC mechanism in removing irrelevant features in the first step is *n*, the time complexity of the maximum information correlation in the second step is *n*, and the time complexity of the recursive feature elimination method in the third step is (*n*/2)^2^, the overall time complexity is (*n*/2)^2^+2*n*. On the CIC-IDS-2017 dataset, the feature selection computation time of the RIC mechanism has increased compared with the MIR mechanism and the CHI mechanism, but it has improved in AR, RR, and F-Score. Compared with the RFE mechanism, the RIC mechanism is greatly shortened in time.

In addition, due to the maximum information correlation feature selection in the RIC feature selection mechanism, compared with the RFE mechanism, the correlation between features and labels can be considered, and the phenotype-related features can be better selected. In AR, RR, F- Score is also better. Therefore, compared with the MIR mechanism, the RFE mechanism, and the CHI mechanism, the RIC feature selection mechanism proposed in this paper can better select the optimal feature subset for network anomaly traffic detection.

### 6.2. Experiment of Network Anomaly Traffic Detection Based on SC-DeCN

In order to verify the effectiveness of the SC-DeCN model proposed in the paper in the detection of network abnormal traffic, experiments were carried out on the CIC-IDS-2017 dataset, using 78 original features after data preprocessing as the input of the model, and combined with the LSTM model, CNN-LSTM model, DSAE model, MSCNN model, and PCCN model are compared experimentally. The AR, RR, and F-Score of the above six network abnormal traffic detection models are shown in Figure 5, and the FAR is shown in Figure 6.

As can be seen from Figures 5 and 6, among the six classification models, the performance indicators of the LSTM model and the DSAE model are lower, so these two models perform poorly in the detection of network abnormal traffic. The variant of the CNN model performs better than other models, among which the MSCNN model performs worse than PCCN and SC-DeCN in all aspects, and SC-DeCN performs best overall. The specific data are shown in Table 3.

In Table 3, compared with the best classification model PCCN in the comparative experiment, the SC-DeCN model has improved by 1.14%, 0.86%, and 0.88% in AR, RR, and F-Score, respectively, and FAR decreased by 0.51%. Among the six classification models, LSTM has the worst classification effect, has not only lower AR but also has the longest model training time.

Although the DSAE model has a short model training time, the AR is too low. The variants of the CNN model, the MSCNN model, and the CNN-LSTM model perform relatively well. Among them, MSCNN has a short training time due to its simple model, but other performances are relatively poor compared to CNN-LSTM. The CNN-LSTM model outperforms the MSCNN model and the LSTM model because it combines the powerful feature extraction capabilities of the CNN model and the LSTM model has certain advantages in dealing with time series problems.

The PCCN model, as a parallel cross convolutional neural network, can extract richer feature information after fusing the branches of the two convolutional neural networks. Compared with the SC-DeCN model, the PCCN model does not perform deconvolution, and its effect in the detection of network abnormal traffic is worse than that of the SC-DeCN model. The experimental results show that the SC-DeCN model proposed in this paper has obvious advantages in the process of abnormal network traffic detection. It can be shown that the information loss problem caused by the pooling operation in the convolutional neural network can be effectively solved by combining the deconvolution model.

### 6.3. Network Anomaly Traffic Detection Based on RIC-SC-DeCN

In order to verify the effectiveness of the combination of the RIC feature selection mechanism proposed in the paper and the SC-DeCN model, the paper uses the SC-DeCN model to conduct comparative experiments, and it is verified on the public dataset CIC-IDS-2017. The experimental results are shown in Table 4.

It can be seen from Table 4 that compared with the SC-DeCN algorithm, RIC-SC-DeCN has an AR increase of 1.13%, RR increased by 1.27%, and F-Score increased by 1.44%. FAR decreased by 1.27% and shortened by 45.50% in time. The experimental results show that the RIC-SC-DeCN model proposed in this paper is better than the SC-DeCN model in the process of network abnormal traffic detection. It can greatly shorten the time used for model training and improve accuracy.

## 7. Conclusions

In the detection of network abnormal traffic, in view of the problem of noise characteristics in network traffic data and the problem of information loss caused by the pooling operation of convolutional neural networks used in existing research, this paper proposes a new method based on RIC-SC-DeCN network abnormal traffic detection algorithm. First, the important features in the network traffic are extracted through the proposed RIC feature selection mechanism, which reduces the impact of noise features and greatly shortens the training time; second, the extraction results are used as the input of the convolutional neural network, automatically learn the deep features of the data; then, combine the deconvolution network to reconstruct the original input signal, and fuse the deep features learned by the convolutional neural network to solve the information loss problem of the pooling operation in the convolutional neural network. The experimental results show that, compared with other classification algorithms, the method proposed in this paper has the best overall performance in terms of accuracy and efficiency.

The maximum information correlation feature selection method used in this paper is unstable in feature selection. In response to this problem, in future research, it can be considered to add stability evaluation criteria to the correlation function, and at the same time, the number of feature subsets and classification error rate indicators are added to the evaluation indicators to form multiobjective evaluation criteria so as to enhance the stability of selecting feature subsets and improve the performance of the network abnormal traffic detection algorithm.

## Figures and Tables

**Figure 1:** The overall framework of the algorithm.

**Figure 2:** SC-DeCN model.

**Figure 3:** Feature selection mechanism experiment comparison.

**Figure 4:** False alarm rate of feature selection mechanism.

**Figure 5:** Anomaly detection performance comparison.

**Figure 6:** Anomaly detection false alarm rate.

**Table 1:** The subset of features selected.

Feature selection	Feature subset
Mechanism	
MIR	2, 11,13, 14, 18, 19, 21, 23, 24, 40, 41, 42, 43, 44, 49, 53, 55, 62, 77, 78
RFE	1, 2, 11, 13, 14, 19, 20, 22, 23, 24, 39, 40, 41, 48, 52, 53, 55, 66, 77, 78
CHI	1, 2, 5, 6, 7, 11, 13, 17, 22, 36, 40, 41, 42, 43, 53, 55, 64, 66, 67, 68
RIC	1, 2, 11, 13, 14, 17, 20, 22, 30, 35, 36, 38, 43, 47, 49, 50, 54, 61, 66, 74

**Table 2:** Comparative experiment of feature selection mechanism.

Method	AR	RR	FAR (%)	F-Score	Feature	Select-time (s)	Model-time (s)	Total-time (s)
	(%)	(%)		(%)				
MIR [6]	93.12	93.08	6.91	93.11	20	78.80	297.17	375.97
RFE [7]	95.57	95.60	4.39	95.61	20	2227.80	295.76	2523.56
CHI [5]	94.13	94.12	5.87	94.13	20	102.09	294.63	396.72
RIC	96.22	96.10	3.89	96.22	20	449.52	298.02	747.54

**Table 3:** Comparative experiment of classification model.

Method	AR (%)	RR (%)	FAR (%)	F-Score (%)	Model-time (s)
LSTM	81.28	81.27	18.72	81.27	1892.07
CNN-LSTM	92.88	92.72	7.27	92.95	2079.37
DSAE	76.79	81.61	18.38	87.95	52.81
MSCNN	91.56	91.49	9.50	91.55	409.78
PCCN	95.41	95.39	4.25	95.40	2014.49
SC-DeCN	96.55	96.25	3.74	96.28	1866.41

**Table 4:** Effectiveness comparison experiment of RIC-SC-DeCN.

Method	AR (%)	RR (%)	FAR (%)	F-Score	Feature number	Select-time (s)	Train-time (s)	Total-time (s)
				(%)				
SC-DeCN	96.55	96.25	3.74	96.28	78	0	1866.41	1866.41
RIC-SC-DeCN	97.68	97.52	2.47	97.72	20	450.79	566.32	1017.11

## Data Availability

All the data used to support the findings of the study are included within the paper.
